The article "Analysis of the Basic Characteristics and Teaching Environment and Mode of Music Appreciation Course Based on Core Literacy" was retracted in 2023. Reasons: unreliable results or conclusions; concerns about the data; concerns about the results or conclusions; concerns about the peer review.

# Analysis of the Basic Characteristics and Teaching Environment and Mode of Music Appreciation Course Based on Core Literacy

**DOI:** 10.1155/2022/7709053

**Published:** 2022-07-31

**Authors:** Hua Lv

**Affiliations:** College of Music, Henan University, Kaifeng 475001, China

## Abstract

The main goals of a music appreciation course are to develop college students' emotions, improve their musical abilities, and strengthen their conceptual framework. This essay primarily introduces the fundamental elements and instructional approach of a music appreciation course built on core literacy. In order to clarify the need for and orientation of basic literacy in college music appreciation teaching, as well as to understand the special value of the subject, we conducted research on the relationship between basic literacy and college music appreciation teaching. Based on this, a new detection algorithm that fuses feature fusion and AM (attention mechanism) is proposed, and visual AM is added to the algorithm based on AM features to help the agent learn the best course of action quickly. The findings indicate that this method's cumulative normalized discount gain increases by about 0.07 and that the recommended list's overall quality has significantly improved. The hit ranking is decreased by about 0.05 when compared to the collaborative neural network filtering method without AM.

## 1. Introduction

Education reform and development in line with China's national conditions have taken the top priority because it serves as a strong foundation for the development of national cultural soft power. As a result, the development of talents has received increasing attention, and education has started, with a focus on developing students' fundamental literacy. College music instruction focuses on the classroom, internalization, and absorption of music knowledge by students, as well as the cultivation, development, and enhancement of students' fundamental musical literacy. Additionally, the new curriculum outlines precise standards and specifications for instructional activities. To allow each student to be the master of their own learning and actively participate in class, various teaching techniques are used for various students and various textbooks [1, 2]. The goal of music curriculum development and reform should always serve as the main driver of appreciation instruction, which is the primary component of music classroom instruction in the fundamental stage. As a result, it is essential to conduct research on music appreciation instruction that is based on fundamental literacy, which is also the general direction of the reform of classroom music instruction in colleges and universities.

Developing students' core literacy has become the focus of educational theory and practice research by countries, educational organizations, and educators all over the world, and the related theoretical and practical research in China is increasing day by day. Mota and Abreu concluded that in the 21st century, when information and knowledge are supreme, core literacy is the ability and moral character that a person should have to deal with problems and quickly adapt to an unfamiliar environment. It not only covers the traditional social vocational skills, but also pays more attention to personal innovation and creativity and communication skills [3]. Turner-Bisset studies music curriculum and thinks that mathematics core literacy can be understood as the comprehensive ability that students should achieve in learning mathematics [4]. Snook et al. and others think that the research from core literacy to subject core literacy is an inevitable choice to promote classroom teaching reform, and the construction of a subject core literacy system must be guided by objective theory, while the way to build subject core literacy must be through the practice of curriculum and teaching [5]. Teachers' immediate evaluation of students in class is also very important. A positive evaluation will make students feel that it is very effective to complete the music guidance plan, which will fill them with a sense of accomplishment and make them like music appreciation class. Then, the significance of using the music guidance plan will be more and more positive.

In colleges and universities, music appreciation classes are one of the key components of the art curriculum. It is crucial to develop college students' ability to appreciate art, but this is more or less accurate when compared to the teaching philosophies, goals, lessons, and methods used in music appreciation classes in colleges and universities. Music education in colleges and universities is not recommended [6, 7]. Students can develop fundamental skills in music appreciation and aesthetics, significantly improve their artistic quality, cultivate their emotions, and improve their personality and quality by appreciating a variety of musical works. This study presents teaching strategies based on feedback from teachers and students, as well as teaching design with specific course examples, all with an emphasis on basic literacy. (1) This study closely monitors the pace of educational reform, curriculum reform, and teaching reform. It conducts teaching research on music appreciation courses using the core literacy reform concept with the goal of finding a teaching activity design method that combines “music-based” and “education-based” to support the implementation of core literacy in the music discipline. (2) Classroom instruction plays a significant role in the overall educational process, and as educational technology advances, more strategies for enhancing the quality of teaching management are made available. A new detection algorithm combining AM and feature fusion is proposed in order to increase the precision of classroom head-up rate detection and strengthen the positive feedback of the teaching situation.

## 2. Related Work

### 2.1. Research on Core Literacy

Basic literacy is defined as the necessary character and key skills that students gradually develop to meet the needs of personal life development and the educational process in the corresponding academic year. This definition comes from relevant theoretical research and educational practice in China. It can be broken down into three main categories: cultural foundation, individual growth, and social engagement. These three categories are represented by six qualities: humanistic inheritance, scientific spirit, learning to learn, healthy lifestyle, sense of responsibility, and practical innovation.

Goudvis and Harvey defined core literacy as a kind of integrated ability, which includes not only individuals' social skills and motivation but also personality characteristics, which determine a person's strength and ability [8]. Schutz and Hoffman pointed out that core literacy should be the moral character and key ability that students should learn and cultivate, which can guarantee their own sustainable development and promote social progress [9]. The core literacy of a discipline is defined as the concrete embodiment of core literacy in a particular discipline, which is the ability and character that students develop imperceptibly after the education, study, and cultivation of the discipline. This ability and character have the characteristics of the discipline, which is generally incapable of being given and cultivated by other disciplines.

Gibson not only clearly defined the cultivation of core literacy but also carefully defined the curriculum content, teaching methods, and evaluation of students. The provisions of the bill also promoted the research of core literacy in this country [10]. Testa and Tonsing take cultivating students' core literacy of different ages as the educational goal, and draw up curriculum objectives and content through core literacy so as to lead the curriculum reform [11]. After research, Wurziger found that in some technology-oriented universities, there are many problems in the training methods of students' comprehensive ability, which leads some universities to attach importance to technology education but neglect the all-around development of students ability [12]. Ebersohnl et al. put forward that the construction of core literacy idea in China should be combined with the specific educational situation, and an education system based on core literacy idea should be established according to the characteristics of social development and students' own development [13]. At the same time, in the process of construction, the relationship between ideas and educational systems should be clearly divided.

### 2.2. Research Status of AM

AM (attention mechanism) [14] is a mechanism that enhances the Encoder + Decoder model's performance by taking into account how people typically observe things. Machine translation was carried out while aligning the source languages, which clearly improved the performance of the neural network machine translation model. In order to alternate collaborative AM on the basis of cascading attention, Hu et al. designed and implemented a dynamic attention network. The iterative process allowed the model to recover from the initial local maximum associated with the incorrect response and produced positive outcomes in the machine reading task of question-answering [15]. In order to apply the Encoder-Decoder framework based on the attention model to the field of speech recognition, Pang S et al. [16] used AM to identify the correspondence between speech and words.

Zheng Z et al. introduced AM to improve the sequence-to-sequence architecture of neural machine translation [17]. After that, it began to be widely used to improve the architectures of various cyclic neural networks and convolutional neural networks [18]. Wang and Wang proposed YOLOv3 algorithm, which uses three-scale feature maps to improve the detection effect of small targets [19]. However, in the classroom video, the characters are relatively complex, feature extraction is difficult, and when students are blocked, it is easy to miss the target. Shi et al. put forward an asynchronous deep reinforcement learning framework, which replaces the traditional experience playback mechanism with the asynchronous method, so that the model does not need to store a large number of training samples, and does not need to extract a small number of samples every time to calculate the loss, thus greatly reducing the storage and calculation expenses [20]. The traditional asynchronous deep reinforcement learning algorithm [21] cannot focus on the visual areas and visual features that are helpful to the final training results, and the introduction of AM will help the learning algorithm effectively solve this problem.

## 3. Methodology

### 3.1. Research on the Basic Characteristics of College Music Appreciation Course Based on Core Literacy

Basic literacy can be implemented successfully in classroom settings. Effective teaching can be completed, which is helpful in the development of fundamental literacy. This involves defining the subject knowledge structure and designing it in the classroom. The author evaluates and synthesizes the works of appreciation that are included in the teaching materials for music, positioning each unit of music appreciation repertoire in every college music appreciation course, as well as the formation trend of the fundamental disciplines of literacy. The genre of works that are liked depends on the students' ages. Genres and forms are expanding and getting richer as students' cognitive levels keep getting better. Students can deepen and broaden their understanding of music aesthetics by learning about the emotions and experiences of various musical genres.

The goal of offering music appreciation courses in colleges and universities is to improve students' capacity for aesthetic appreciation through listening to, feeling, understanding, and understanding music. It also aims to introduce college students' musical cultural backgrounds through music appreciation so that they can learn about stories. The importance of the times, the composer's studies, and the composer's creative heritage all have a greater influence on his future professional success. Music has the qualities of moral education, and its social and educational benefits cannot be disregarded. The engine and source of human society's advancement and development is innovation. The potential and creativity of students are greatly enhanced and fostered by music. Because listening is directly related to the level of music appreciation and because listening more can enhance listening and support memory, the development of sensitivity must also include the development of students' listening skills. School administrators spend a lot of time in the classroom guiding teachers' practice and postlesson reflection; well-known educators and up-and-coming educators assist and mentor students in the classroom. Throughout the academic year, we will conduct group research classes and engage in activities to hasten the development of teachers' classroom teaching skills at various levels.

The intrinsic value of educating people and the importance of choosing social talents are two value orientations of the current curriculum evaluation system, both of which are set against the backdrop of basic literacy. These two values are distinct and at odds with one another, which is the fundamental issue. Education becomes a by-product of choice when teaching and learning are done for the sake of choice. Students from various majors can select programmes based on their own characteristics after a platform has been established for them, which not only helps them to improve the quality of their own music but also serves as an example for other students to follow and learn from by sharing knowledge with one another. Teachers need to focus more on the interests and personalities of their students every day. Though some music educators might disagree, this does relate to music lessons. Students' motivation to learn music will increase if their performance is more accurately assessed and they are given encouragement.

The new music curriculum standard is a programmatic guiding document for the implementation of music teaching, and its ideas and requirements guide the practice of music education and teaching. The value of music education includes the value of music noumenon and the value of music nonnoumenon. The value of music noumenon refers to the musical ability, skills, perception, and musical thoughts acquired around music learning. The nonontology value of music refers to the acquisition of music through music learning. Discipline teaching is the carrier of the ultimate practice of basic literacy. The specific operation form and practice of basic literacy need to be supported by specific teaching practices. The basic characteristics of a college music appreciation course based on core literacy are shown in Figure 1.

Based on the above understanding, the idea of school curriculum system construction is to do a good job in the integration and reorganization of the national curriculum, local curriculum, and school-based curriculum, and combine them into one to implement and design the school curriculum system. Taking the curriculum as a whole and the development of students' basic literacy as the core, giving students enough rights to choose courses that they are interested in, and leaving room for their future development is also the idea of implementing checkpoint design in schools.

Therefore, to understand the basic literacy, we must first study this comprehensiveness. Only by deeply understanding the concept of basic literacy can we understand the leading role of basic literacy, provide directions for the reform research of various disciplines, and highlight its leading role. When emphasizing the basic qualities necessary for cultivating talents, we should not ignore the value and function of knowledge. The process of knowledge formation is also the process of quality cultivation. Teachers should understand that music knowledge is not only a carrier but also an aid, so it is naturally not the main body of teaching. When designing and organizing classroom teaching activities, teachers must accurately understand the relationship between music knowledge and the role that music knowledge should play.

The ability to practice music is the key and difficult point to cultivate in students with basic musical literacy, and the perception and understanding of musical works is a spiritual experience. The process of improving music appreciation ability and music aesthetic ability is the process of upgrading auditory experience to spiritual experience. Musical aesthetic ability is the transition from the level of people's emotional expression of music to the level of understanding the thoughts and emotions expressed by music. After appreciating the works, students should have a spiritual experience of the works, that is, music aesthetics. College music appreciation course is developed through music appreciation and music aesthetics. In this process, students' ability to appreciate music is improved, and students' musical literacy is improved.

### 3.2. Design of the Teaching Mode Based on Core Literacy

Male and female beauty are two categories of aesthetics. Comedy beauty and tragic beauty are two categories of emotional development. It is necessary to establish a music appreciation class because it is not only one of the crucial tools for aesthetic education but also the best example of moral education. Men's works include those that depict the conflict between man and nature and fate, which can strengthen people's will. People use music as a way to express their inner feelings and understanding of musical works by fusing their interest in music, artistic forms of music, and emotional experience of music. As opposed to mass producing and assembling products, teachers should always approach their students with a positive attitude and a developmental perspective. They should also believe in, respect, and believe that students have limitless potential.

The introduction of background information aids students in understanding the connotation and level of music they hear and aids in their discovery of beauty when teaching music appreciation. In order to ensure that students accurately understand the connotation of the works and experience their profound vitality, it is crucial to introduce background cultural knowledge when teaching students to appreciate musical works. It is more crucial to popularize and comprehend background cultural knowledge when learning music that has overtly ethnic or national characteristics. A student's ability to appreciate music can be improved, which can encourage the development of the discipline's basic literacy and ultimately lead to the realization of basic literacy. The proper introduction of prior musical knowledge is of positive significance in enhancing music experience and aesthetic ability.

In the subject-based classroom, students must actively participate in all teaching activities [8]. Teaching means teachers and students participate in classroom discussions, promote the transfer of learning according to students' experience and foundation, and cultivate students' ability to solve problems and think ahead. Generally speaking, the overall design of subject teaching can be divided into three stages: preliminary preparation, development and design, and evaluation and revision, which may include the following steps, as shown in Figure 2.

Teaching design often involves different learning stages, so in teaching, we should carefully divide different contents according to the specific situation. In teaching design, we should pay full attention to students' existing learning experience, students' learning characteristics, characteristics of music courses, etc., so that students can explore and find solutions to problems in activities and modes. AM is one of the research hotspots of deep learning in computer vision, natural language processing, speech recognition, and other fields. AM can help the learning model shift its attention to the input parts that deserve attention, instead of balancing each input data and then extracting the best information features. Calculation of the weight coefficient of each area pixel by softmax function:

(1) $$\begin{array}{c} a_{ti}=\frac{\exp\left(e_{ti}\right)}{\sum_{k=1}^{L}\exp\left(e_{ti}\right)}, \end{array}$$

where *L* represents the number of regional pixels of the image.

The user feature set and music feature set are obtained as vectorized representations after being separately input into the word embedding layer. The user set is shown as

(2) $$\begin{array}{c} U=\left\{u_{1},u_{2},\ldots ,u_{m}\right\}. \end{array}$$

Among them, *u*_*i*_=∑_*m*_*u*_*f*_.

The user feature set is represented as

(3) $$\begin{array}{c} u_{f}=\left\{u_{f1},u_{f2},\cdots ,u_{fm}\right\}. \end{array}$$

The music collection is represented as

(4) $$\begin{array}{c} M=\left\{m_{1},m_{2},\ldots ,m_{N}\right\}. \end{array}$$

Among them, *m*_*j*_=∑_*n*_*m*_*f*_.

The music feature set is represented as

(5) $$\begin{array}{c} m_{f}=\left\{m_{f1},m_{f2},\ldots ,m_{fn}\right\}. \end{array}$$

The feature *U*_*f*_ of each user and the feature *M*_*f*_ of each piece of music are obtained through the fully connected network. The user's preferred function for music features, namely, attention, can be learned by AM:

(6) $$\begin{array}{c} a_{ij}=\tanh\left(w_{ij}h_{m_{j}}+b_{ij}\right), \end{array}$$

where {*h*_*m*_1__, *h*_*m*_2__,…, *h*_*m*_*n*__} is the hidden layer state value corresponding to the music feature set {*m*_*f*_1__, *m*_*f*_2__,…, *m*_*f*_*n*__}, *w*_*ij*_, *b*_*ij*_ is a parameter obtained through model training, *w*_*ij*_ represents the weight of user *u*_*i*_ to the *j* th feature of music *m*_*k*_, and *b*_*ij*_ represents the offset.

For this model, we also use *L*_2_ norm for regularization, which is a common technique in machine learning, aiming at reducing the complexity of the model by limiting the weight. This is done by adding a weight penalty to the cost (loss) function:

(7) $$\begin{array}{c} C_{\text{final}}\;\left(\hat{Y},Y\right)=C\left(\hat{Y},Y\right)+\gamma \frac{1}{n}\sum_{i=1}^{n}w_{i}^{2}. \end{array}$$

Where $C\left(\hat{Y},Y\right)$ is the loss (cost) function of network output $\hat{Y}$ and expected output *Y*, and *w*_*i*_ is the learnable weight in the network. The final cost function increases with the increase in weight so that the model with a larger weight in the network is punished. In order to normalize the model, it is necessary to adjust the probability value of dropout and the attenuation factor of *L*_2_ norm regularization.

Hollow convolution can enlarge the receptive field and filter redundant features. The essence of convolution is the extension of general convolution, and its output *y*[*i*] can be expressed as

(8) $$\begin{array}{c} y\left[i\right]=\sum_{k=1}^{k}x\left[i+r\times l\right]w\left[l\right], \end{array}$$

where *x* [·] represents a one-dimensional input signal; *w*[*l*] is convolution kernel; *l* is the convolution kernel size; and *r* is the expansion coefficient.

Information flows only in one direction, that is, the output of each layer is only determined by the output of the previous layer. This constraint makes it easy for the neural network to realize computational training and reasoning through basic linear algebra operations. We can use the following formula to represent the hidden layer:

(9) $$\begin{array}{c} H=f\left(b+X*W\right). \end{array}$$

Here, *X* ∈ *R*^1×3^, *W* ∈ *R*^4×6^, *H* ∈ *R*^1×5^. The weighted sum of neurons in each hidden layer can be calculated by using a single-matrix multiplication. It is very fast to run such a large number of matrix and vector calculations on the GPU.

The structure of the head-up rate detection algorithm based on AM and feature fusion is shown in Figure 3.

Compared with the human face, the head contains more visual information and is less affected by occlusion, which plays an important role in the detection of head-up rate. The input features are processed by the channel attention module and the spatial attention module in turn, and the refined features are obtained. In classroom video, the classroom background and objects are not the focus of attention, so adding an attention model to the network can improve the ability to extract effective features. After the header bounding box set is obtained, the thinning module is used to further refine the results.

## 4. Experiment and Results

Asynchronous deep reinforcement learning replaces the traditional experience playback mechanism with multithreading technology, which not only solves the correlation between training samples but also speeds up the training time of learning model. In order to effectively verify the learning performance of this model, this chapter compares its performance in the game. The training process is shown in Figure 4.

It can be seen that in the process of game training, the training performance of model in ref [17] in the initial stage is obviously better than that of this model. However, with the increase of training stage, the training effect of this method gradually reaches the level of reference [17], and even in the later stage, it far exceeds the learning performance of ref [17]. The asynchronous actor-critic algorithm with dual AM has better game learning performance than other algorithms, which proves that dual AM can help the model process the game state information more accurately so that the agent can make the best decision faster and more effectively.

Hit ranking is a metric that can be used to gauge how well the recommendation results are performing in real time by determining whether the songs that users have listened to are among the top 10 on the recommendation list. The output of AM is the user's interest weight vector, which represents the user's recent behaviour preference of listening to music. Recent user interest models are highly pertinent, and the recommendation is real time. By working out the formula, we can generate a music vector that is similar to the user's interests, create a list of recommended songs, and create individualized music recommendations for particular users. Hit level value and normalized discount cumulative gain for each algorithm are contrasted in Figures 5 and 6, respectively.

The normalized discount cumulative winning index value has increased and the hit ranking value obtained by this method has decreased when compared to the previously advised method, indicating an improvement in these two indices over the old algorithm. The normalized discount cumulative gain of this method among them is up about 0.07 in comparison to reference [16] method, and the recommended list's overall quality has significantly improved. The hit ranking is decreased by about 0.05 when compared to the collaborative neural network filtering method without AM.

The user interest model created has better representational capabilities thanks to the integration of a variety of user features, music features, and music information, which can help solve the issue of data scarcity. By combining natural language processing technology to process music names and music labels, the feature information of the source data can be better obtained. Add AM to the model to make the recommendation result more understandable. This demonstrates the value of incorporating AM into deep learning, which helps to increase recommendation accuracy and decrease computational complexity. Figures 7 and 8 contain summaries of all experimental results of two data sets. For all neural network models, we report the average precision, recall rate, F1 score, and accuracy rate of the models. We focus on the above four indicators because they show the general performance of the sentiment analysis model.

Our results show that the overall performance of the self-service network is better. Using the same word embedding, all self-care models achieve higher accuracy than all reference models. This paper model usually performs best for all combinations (input insertion and data sets) and gets the highest score in one of the two data sets. In order to simplify our training process and improve efficiency, we decided not to modify the learning rate specifically for each input word embedding dimension. Here, we compare the training and testing efficiency, memory consumption, and the number of trainable parameters of each model. For all models, we use data set 1 as an intuitive example, with a hidden size of 300 and a batch size of 32 for training and reasoning.  Table 1 contains a summary of the characteristics of the model.

The model in ref [16] has the least number of parameters but consumes the most GPU memory. Because there are fewer parameters to be trained, it also has the shortest training and reasoning time. Compared with model in ref [19], the number of parameters of model in ref [20] is twice that of our method, and the training and reasoning time is almost twice that of our method. This is reasonable because both architectures have two AM layers.

Table 2 shows the performance comparison between the feature fusion attention rate detection algorithm and other attention rate detection algorithms in the data set. The calculation time is the time taken to detect a 15-second video clip with a frame rate of 25 frames per second. Although the algorithm proposed in this paper is based on deep learning, the speed is slightly slower, but it has achieved good performance in accuracy, and the error is only about 15%.

After AM, the output result is the user's interest preference vector, which depicts the user's interest preference model of recent musical listening. To obtain the user interest weights of various music feature vectors and the interest weights of each song in the history list, deep learning is applied to a variety of source data, with the feature set and the music itself serving as the minimum processing units. The user weight is then updated. It is beneficial to reduce the issue of data scarcity, enhance the real-time functionality of recommendation systems, and get more precise recommendation results.

In order to help students discover, feel, and experience beauty and to improve their capacity to feel and appreciate in subtle ways, students are given music knowledge through situational teaching in vivid settings. Real-world situations can construct life situations, problems, images, etc., as well as create situations for students from the perspectives of actions and new and old knowledge. There are many different types of situations. It enables students to make connections between their past experiences and the subject matter they are currently learning, allowing knowledge to pass through the experience gap and become practical knowledge, transforming them into the main component of the classroom. In order to more effectively accomplish the objective of “cultivating students under the guidance of basic literacy,” knowledge learning and implementation are necessary.

In addition to having a basic understanding of music theory and being able to play an instrument, students who lack basic music literacy must work on developing their aesthetic and cognitive understanding of music. The teacher can introduce the lesson plans and outside resources when he serves as the host. The main goal of the specific instruction is to motivate learners to seek answers or direct learners to attempt problem-solving independently. Teachers will explore the mysteries in great detail and broaden their students' knowledge after assisting them in learning more about the issues as they work to solve. Overseeing is the responsibility of teachers. It should be noted that this method of instruction is not meant to be used throughout the entire class or for the duration of the thematic courses that are being taught in the group.

## 5. Conclusions

The ability to appreciate music is not only one of the important symbols of aesthetic achievement but also its educational function for students cannot be replaced by any other teaching method. Starting from the demand and orientation of basic literacy for music appreciation teaching, this paper studies the interactive relationship between appreciation teaching and basic literacy, forms a map of demand and orientation, and the implementation path of basic literacy in music appreciation teaching. In order to improve the quality of classroom supervision and management, this paper proposes a class head-up rate detection algorithm combining AM and feature fusion. The experimental results show that the cumulative gain of the normalised discount of this method is increased by about 0.07, and the overall quality of the recommended list is greatly improved. Compared with the collaborative neural network filtering method without AM, the hit ranking is reduced by about 0.05. We have achieved better model functions, such as lower memory consumption, faster training/reasoning time, and fewer trainable parameters.

## Figures and Tables

**Figure 1:** Appreciating the basic characteristics of music courses.

**Figure 2:** Theme teaching design.

**Figure 3:** Algorithm structure.

**Figure 4:** The training process in the game.

**Figure 5:** Comparison of hit ranking values of algorithms.

**Figure 6:** Comparison of normalized discount cumulative gain of algorithms.

**Figure 7:** Result presentation of data set 1.

**Figure 8:** Result presentation of data set 2.

**Table 1:** Characteristics of neural network architecture.

Model	GPU memory (MB)	Trainingtimes	Reasoningtimes
Methods of this paper	380	66.2	8.27
Ref [16]	988	20.33	0.86
Ref [19]	421	233.61	7.71
Ref [20]	701	415.28	15.24

**Table 2:** Performance comparison of different head-up rate detection algorithms on data sets.

Model	Error/%	Run time/s
Methods of this paper	15.326	50.271
Ref [16]	19.661	33.025
Ref [19]	20.103	28.906
Ref [20]	16.025	66.821

## Data Availability

The data used to support the findings of this study are available from the author upon request.

## References

[1] Zeyer A., Cetin-Dindar A., Md Zain A. N., Jurisevic M., Devetak I., Odermatt F. (2013). Systemizing: a cross-cultural constant for motivation to learn science. *Journal of Research in Science Teaching*.

[2] Petchauer E. I. (2011). I feel what He was doin. *Urban Education*.

[3] Mota G., Abreu L. (2014). Thirty years of music and drama education in the Madeira Island: facing future challenges. *International Journal of Music Education*.

[4] Turner-Bisset R. (2010). Serving-Maids and Literacy: an approach to teaching literacy through history and music. *Literacy*.

[5] Snook A. G., Schram A. B., Jones B. D. (2021). Faculty’s attitudes and perceptions related to applying motivational principles to their teaching: a mixed methods study. *BMC Medical Education*.

[6] Chen C. (2022). Design of deep learning network model for personalized music emotional recommendation. *Security and Communication Networks*.

[7] Ramos K. (2014). Teaching adolescent ELs to write academic-style persuasive essays. *Journal of Adolescent & Adult Literacy*.

[8] Goudvis A., Harvey S. (2012). Teaching for historical literacy. *Educational Leadership Journal of the Department of Supervision & Curriculum Development N.e.a*.

[9] Schutz K. M., Hoffman J. V. (2017). “I practice teaching”: transforming our professional identities as literacy teachers through action research. *The Reading Teacher*.

[10] Gibson S. J. (2021). Shifting from offline to online collaborative music-making, teaching and learning: perceptions of Ethno artistic mentors. *Music Education Research*.

[11] Testa E., Tonsing C. S. (2014). Kindle-ing the common core. *Journal of Adolescent & Adult Literacy*.

[12] Wurziger J. (2010). Reading teachers’ learning/teaching styles: keys to effective supervision and evaluation. *Literacy*.

[13] Ebersoehn L., Joubert I., Prinsloo Y., Kriegler S. (2014). Outcomes of an English literacy intervention on non-mother tongue teaching practices of teachers in rural schools. *Value in Health*.

[14] Li M., Zhou G., Cai W. (2022). Multi-scale sparse network with cross-attention mechanism for image-based butterflies fine-grained classification. *Applied Soft Computing*.

[15] Hu J., Yan P., Su Y., Wu D., Zhou H. (2021). A method for classification of surface defect on metal workpieces based on twin attention mechanism generative adversarial network. *IEEE Sensors Journal*.

[16] Pang S., Zhang Y., Song T., Zhang X., Wang X., Rodriguez-Paton A. (2022). AMDE: a novel attention-mechanism-based multidimensional feature encoder for drug–drug interaction prediction. *Briefings in Bioinformatics*.

[17] Zheng Z., Liu Y., He M., Chen D., Sun L., Zhu F. (2022). Effective band selection of hyperspectral image by an attention mechanism-based convolutional network. *RSC Advances*.

[18] Chen L., Shi W., Deng D. (2021). Improved YOLOv3 based on attention mechanism for fast and accurate ship detection in optical remote sensing images. *Remote Sensing*.

[19] Wang W., Wang J. (2021). Double ghost convolution attention mechanism network: a framework for hyperspectral reconstruction of a single RGB image. *Sensors*.

[20] Shi C., Zhao X., Wang L. (2021). A multi-branch feature fusion strategy based on an attention mechanism for remote sensing image scene classification. *Remote Sensing*.

[21] Huang Y., Cheng L., Xue L. (2021). Deep adversarial imitation reinforcement learning for QoS-aware cloud job scheduling. *IEEE Systems Journal*.

